This article has been retracted.

# Effectiveness of “Internet+” Based Cardiac Rehabilitation on Prognosis of Patients with Coronary Heart Disease: A Meta-Analysis

**DOI:** 10.1155/2022/1574774

**Published:** 2022-05-20

**Authors:** Meng Ding, Fan Zhang, Jiashun Hu

**Affiliations:** ^1^Department of Operation Room, Wuhan Hankou Hospital, Wuhan, Hubei 430012, China; ^2^Department of Information Centre, Wuhan Hankou Hospital, Wuhan, Hubei 430012, China; ^3^Department of Internal Medicine-Cardiovascular, Wuhan Hankou Hospital, Wuhan, Hubei 430012, China

## Abstract

**Objective:**

Meta-analysis was used to systematically evaluate the impact of Internet-based cardiac rehabilitation on the health of patients with coronary heart disease.

**Methods:**

Randomized controlled trial study (RCTs) of the effects of Internet-based cardiac rehabilitation on cardiovascular risk factors, motor function and psychological status in patients with coronary heart disease has been systematically studied.

**Results:**

A total of 13 articles were included. Meta-analysis showed that internet-based cardiac rehabilitation training could effectively reduce the total cholesterol level [MD = -0.15, 95% CI (-0.28, -0.02), *P* = 0.02] and triglyceride level [MD = -0.19, 95% CI (-0.32, -0.06), *P* = 0.01], increase the maximal oxygen uptake (VO2 max) [MD = 0.9995, CI (0.161.83) *P* = 0.02] and physical activity level [SMD = 0.51, 95% CI (0.07, 0.9), *P* = 0.02], and improve the self-efficacy [SMD = 0.50, 95% CI (0.17, 0.83), *P* = 0.01] and improved quality of life [SMD = 1.34, 95% CI (0.12, 2.56), *P* = 0.03] of patients. However, there was no significant improvement in blood pressure and body mass index, depression and anxiety.

**Conclusion:**

Internet-based cardiac rehabilitation can significantly reduce cholesterol and triglyceride levels and improve theVO_2_ max, physical activity, self-efficacy and quality of life, but is not effective on the level of blood pressure, BMI, anxiety and depression. Due to the limitations of methodological quality and sample size of included studies, more studies with high-quality and large sample are needed to further evaluate its effectiveness.

## 1. Introduction

With the improvement of people's living standard and the change of diet structure, the incidence of coronary heart disease (CHD) increased year by year. The number of cardiovascular patients in China has exceeded 330 million, among which coronary heart disease has exceeded 11 million and is increasing by 20% every year [1]. At present, surgery and drug therapy cannot completely eliminate the risk factors of coronary heart disease, and patients still need to recover cardiopulmonary function through rehabilitation training [2, 3]. Cardiac rehabilitation is a comprehensive intervention method, including guiding patients to take medicine regularly and exercise training and guiding their diet and health education, which is an important means to reduce the incidence and sudden death rate of patients with coronary heart disease and improve the quality of life of patients [4, 5]. Although the model of cardiac rehabilitation has been established, due to the limitations of time and environment, the development of cardiac rehabilitation is not ideal, and patients' participation and exercise duration are low [4, 6]. Internet + refers to the provision of medical information and services through communication technology, which has been widely used in many fields such as disease prevention, chronic disease self-management and health promotion [7]. Although there has a been meta-analysis of the effects of Internet+ based cardiac rehabilitation on CHD patients' health, this analysis did not include studies of China [8]. Therefore, this study aims to evaluate the impact of Internet + based cardiac rehabilitation on the health of patients with coronary heart disease through a systematic search of Chinese and English literatures and provide medical evidence for its promotion and application.

## 2. Materials and Methods

### 2.1. Retrieval Strategies

The Chinese and English literatures published from the establishment of the relevant database to March 2021 were searched, excluding the grey literatures not published publicly. The English subject words, titles and keywords “Internet OR online OR website OR mobile application OR APP OR telemedicine or telehealth OR ehealth OR digital health OR mobile health OR mhealth OR Wechat AND Coronary heart disease OR heart disease OR angina pectoris OR myocardial infarction OR coronary stent implantation OR percutaneous coronary intervention OR percutaneous coronary stent implantation OR coronary artery bypass AND cardiac rehabilitation” were used to retrieve the databases of PubMed, Web of science, Cochrane library, Embase and EBSCO. The Chinese titles and keywords “Internet OR telemedicine OR mobile health care OR mobile phone OR application program OR WeChat AND coronary heart disease OR angina OR myocardial infarction OR percutaneous coronary intervention OR percutaneous coronary stent implantation OR bypass operation of coronary artery AND cardiac rehabilitation OR cardiovascular rehabilitation” were used to retrieve the China National Knowledge Internet (CNKI), Wanfang Database and VIP database. Further search was carried out by the obtained references, similar literatures and related literatures.

### 2.2. Literature Inclusion and Exclusion Criteria

#### 2.2.1. Literature Inclusion Criteria

(1) Study type: Randomized controlled trial (RCT); (2) Intervention population: Adults diagnosed with coronary heart disease (atherosclerosis, angina, myocardial infarction) or coronary revascularization; (3) Intervention methods: Routine nursing was carried out in the control group, and “Internet+” based cardiac rehabilitation or “Internet+” based cardiac rehabilitation based on control group was carried out in the experimental group. (4) Outcomes: Cardiovascular risk factors (blood pressure, body mass index (BMI), cholesterol), motor function indicators (V_O2_ Max, physical activity), and mental health indicators (quality of life, anxiety, depression, self-efficacy)

#### 2.2.2. Literature Exclusion Criteria

(1) The articles with data that were not related to this study or cannot be converted to the required data; (2) Repeatedly published papers; (3) Low-quality literature; (4) Case report, Reviews, abstracts, conference papers; (5) Unable to get full text; (6) Incomplete data or data error; (7) Literature other than Chinese and English

### 2.3. Literature Screening and Data Extraction

Two researchers independently evaluated the included articles. The data of the included literature shall be extracted and resolved through negotiation when there is divergence. The data extracted included first author, characteristics of study subjects, sample size, intervention measures and outcome indicators. Finally, the formal data table (Table 1) was formed after discussion between the two people.

### 2.4. Literature Quality Evaluation

The quality of the articles was assessed by two trained researchers using the bias assessment tool of Cochrane Handbook for Systematic Review of Interventions 5.1.0. The evaluated contents included random sequence generation, allocation concealment, blind method, description of lost follow-up, selective reporting of study results, and other sources of bias.

### 2.5. Statistical Analysis

Meta-analysis was performed on the data by Revman 5.3 software. Mean difference (MD) or standardized mean difference (SMD) were used as the effect indicator. Heterogeneity between studies was determined by Q test. When I^2^>50% and *P* ≤0.1, subgroup analysis or sensitivity analysis was used to determine the source of heterogeneity or only descriptive analysis was performed. If heterogeneity could not be eliminated, random effect model was used to combine effect size. When I^2^<50% and *P* >0.1, it can be regarded as no heterogeneity and fixed effect model was used for analysis.

## 3. Results

### 3.1. Retrieved Results

A total of 1,168 related articles were retrieved. Among them, 133 were in Chinese and 1,035 were in English. By Noteexpress software processing, 897 duplicate articles were deleted. After reading the titles and abstracts of the articles, 235 articles that did not meet the standards were included. After searching for the full text and reading the whole article, a total of 13 articles were finally included. Literature screening process is shown in Figure 1.The basic characteristics and quality evaluation of the included studies are shown in Table 1.

### 3.2. Results of Meta-Analysis

#### 3.2.1. Influence of Internet + Cardiac Rehabilitation on Patients' Blood Pressure

Nine articles [9–13, 17–20] reported the effect of “Internet +” based cardiac rehabilitation on blood pressure of patients with coronary heart disease. Nine of these articles [9–13, 17–20] reported data on systolic blood pressure, and eight articles [9–11, 13, 17–20] reported on diastolic blood pressure. Combined analysis on systolic blood pressure showed relatively large heterogeneity (*P* <0.05, I^2^ = 84%). The random effect model showed no statistically significant difference between the two groups [MD = -0.03, 95% CI (-5.12, 5.06), *P* = 0.99] (Figure 2). Combined analysis on diastolic blood pressure showed relatively small heterogeneity (*P* = 0.28, I^2^ = 18%). The fixed-effect model showed no statistically significant difference between the two groups [MD = -1.03, 95% CI (-2.61, 0.55), *P* = 0.20] (Figure 3).

#### 3.2.2. Influence of Internet + Cardiac Rehabilitation on BMI of Patients

Six literatures [9, 10, 12, 16–18] reported the effect of “Internet +” based cardiac rehabilitation on BMI of patients with coronary heart disease. The heterogeneity was small (*P* = 0.85, I^2^ = 0%). The fixed-effect model results showed no statistically significant difference between the two groups [MD = 0.00, 95% CI (-0.35, 0.35), *P* = 0.99] (Figure 4).

#### 3.2.3. Influence of Internet + Cardiac Rehabilitation on Blood Lipid of Patients

Nine articles [9, 10, 12, 16–20] reported the effect of “Internet +” based cardiac rehabilitation on total cholesterol, with a total of 1,109 subjects included. The heterogeneity was small (*P* = 0.13, I^2^ = 37%). The results of fixed-effect model showed that there was statistically significant difference in cholesterol reduction between the two groups [MD = -0.15, 95% CI (-0.28, -0.02), *P* =0.02] (Figure 5).

Seven articles [9, 12, 17–20] reported the effect of “Internet +” based cardiac rehabilitation on triglyceride, with a total of 925 subjects included. The heterogeneity was small (*P* = 0.86, I^2^ = 0%). The results of fixed-effect model showed that the decrease degree of triglyceride in the experimental group was significantly different from that in the control group [MD = -0.19, 95% CI (-0.32, -0.06), *P* = 0.005] (Figure 6).

#### 3.2.4. Influence of “Internet +” Based Cardiac Rehabilitation on Other Outcome Indicators of Patients (Table 2)

Four literatures [9, 13, 16, 17] reported the effect of cardiac rehabilitation based on “Internet +” on maximal oxygen uptake in patients with coronary heart disease. The heterogeneity was small (*P* = 0.27, I^2^ = 23%). The results of fixed-effect model showed that the improvement degree of maximal oxygen uptake in the experimental group was significantly different from that in the control group [MD = 0.99, 95% CI (0.16, 1.83) *P* =0.02].

In addition, 4 literatures [11, 12, 18, 21] reported the influence of “Internet +"based cardiac rehabilitation on physical activity of patients. Six-minute walking experiment [12, 21], metabolic equivalent [18] moderate amount of physical activity [11] were used for evaluation. It was found that difference between the two groups was statistically significant [SMD = 0.51, 95% CI(0.07, 0.9), *P* =0.02].

Four literatures [11, 14, 17, 19] reported the impact of “Internet +” based cardiac rehabilitation on quality of life of patients. The heterogeneity was large, so the random effect model was adopted. MacNew Scale [11, 14], Dartmouth Quality of Life [17] and Chinese Cardiovascular Patients Quality of Life Assessment Questionnaire [19] were used to assess the quality of life in the four literatures. Due to the different scales of evaluation, the standardized mean was adopted, and the results showed statistically significant differences between the two groups [SMD = 1.34, 95% CI (0.12, 2.56), *P* = 0.03].

Three studies [11, 14, 18] reported the impact of “Internet +” based cardiac rehabilitation on self-efficacy of patients. General self-efficacy scale [11, 14] self-designed questionnaire [18] were used for evaluation. The heterogeneity was small, so the fixed effect model was adopted. The results showed that there was significant difference between the two groups [SMD = 0.50, 95% CI (0.17, 0.83), *P* = 0.01].

Six articles [10–12, 14, 16, 19] reported the effects of Internet + based cardiac rehabilitation focus on depression. Hospital Anxiety and Depression Scale (HAD) [10, 11, 14, 16], Patient Health Questionnaire-9 (PHQ-9) [12], Generalized Anxiety Disorder-7 scale (GAD-7) [12] and Somatization Symptom Self-Rating Scale [19] were used for evaluation. he results showed no statistically significant difference between the two groups.

### 3.3. Publication Bias and Sensitivity Analysis

Funnel diagram was plotted for the influence of Internet+ cardiac rehabilitation on diastolic blood pressure of patients with coronary heart disease, and the results showed that the two groups were symmetrical with no obvious publication bias, as shown in Figure 7. The fixed-effect model and random effect model were used to analyze each model, and the results of effect size were similar, indicating that the meta-analysis had stable and reliable quantitative combined results.

## 4. Discussion

### 4.1. Effect Evaluation of Internet+ Based Cardiac Rehabilitation

Maximal oxygen uptake and physical activity are important indexes to evaluate exercise tolerance of coronary heart disease. Many evidence-based medical evidences show that low level of exercise function is closely related to the risk of cardiovascular disease and all-cause mortality [22–24]. Prospective studies [25] also found that triglyceride levels were significantly positively correlated with the risk of coronary heart disease. However, the lack of supervision of home cardiac rehabilitation often leads to insufficient exercise of patients, and the intervention effect cannot be guaranteed [5]. This study found that cardiac rehabilitation based on Internet + can increase activity tolerance and reduce total cholesterol and triglyceride levels of patients, and the results are similar to Su [8] and Rawstorn et al. [26] In the study of Rawstorn et al. [26], physical exercise level of patients undergoing home cardiac rehabilitation based on electronic technology was superior to patients receiving routine home rehabilitation or routine nursing, but there was no significant difference in aerobic exercise capacity between the two groups of patients in their study [26]. In the study, there was no significant difference in aerobic exercise capacity between the two groups, and the study combined two indicators of maximal oxygen uptake and metabolic equivalent, which showed large heterogeneity and may have some bias. In the present study, the reasons for the heterogeneity of physical activity may be related with the different subjects and measurement time, but the random effect model showed that the physical activity of the experimental group was improved compared with that of the control group. Cardiac rehabilitation training based on Internet + mode is more accessible, and continuous remote nursing monitoring is conducive to timely understanding of patients' lifestyle and providing professional support, enhancing exercise effects and promoting patients' recovery.

In addition, this study found that cardiac rehabilitation based on Internet + could enhance patients' self-efficacy and improve their quality of life. Su et al. [8] also reported in their meta-analysis that cardiac rehabilitation training can improve patients' quality of life. Some intervention studies [11, 12, 15] adopted the comprehensive cardiac rehabilitation model to emphasize the addition of lifestyle management on the basis of exercise and enhanced the support for cardiac rehabilitation of patients by combining team support and real-time supervision of online courses. At the same time, combined with theories such as planned behavior theory or cognitive behavior theory [4, 11], positive feedback is provided to patients in the form of behavioral feedback and empowerment. These measures were likely to improve patients' sense of self-efficacy. The beneficial process or result of intervention further improved their quality of life. Therefore, it is expected to further strengthen the intervention effect to develop a comprehensive cardiac rehabilitation program based on exercise.

This study found that Internet + cardiac rehabilitation did not significantly improve patients' blood pressure, BMI, anxiety and depression and other indicators, which may be related to the different forms, frequency, duration and intensity of exercise. Besides, BMI, systolic blood pressure and other indicators have large individual differences, which are not sufficient for significant changes in a short term. More studies are needed in the future to evaluate the long-term effects of Internet-based cardiac rehabilitation on patients' psychological and long-term cardiovascular events.

### 4.2. Methodological Quality Evaluation of Included Studies

Of the 13 included studies, 3 were of grade A quality, 10 were of grade B quality, and 10 described scientific randomization methods, indicating that the results were credible. In the included literature, only 6 studies implemented concealed grouping. Since the intervention process of Internet + cardiac rehabilitation requires the cooperation of patients and the guidance of experimenters, it is difficult to blind the interveners. Therefore, implementation bias was inevitable. However, blind method was applied to outcome measurement in some studies, and most outcome indicators were objective measurement indicators, thus avoiding measurement bias to a certain extent. All included literatures explained the situation of loss of follow-up and withdrawal, with good data integrity.

### 4.3. Limitations

Heterogeneity existed in the study sample and methodology, such as different forms, frequency and duration of intervention of cardiac rehabilitation. Individual patient differences and limited feasibility of blind implementation were also part of the factors leading to heterogeneity. This paper focuses on the effect of Internet + cardiac rehabilitation on patients with coronary heart disease. Although there was high heterogeneity among some results of the study, it also revealed the necessity of this study from the side. In this study, only Chinese and English literatures were included, and literatures in other languages were not searched, which may lead language bias.

## 5. Summary

Compared with conventional rehabilitation, Internet + cardiac rehabilitation can effectively improve exercise tolerance, reduce blood lipid levels and improve the quality of life of patients with coronary heart disease, but the effect on blood pressure, BMI and other cardiovascular factors is not clear. Due to the limitations of the number and quality of the included studies, more high-quality studies are needed to validate it.

## Figures and Tables

**Figure 1:** Flowchart of the Literature screening process.

**Figure 2:** Influence of Internet+ based cardiac rehabilitation on systolic blood pressure of patients with coronary heart disease.

**Figure 3:** Influence of Internet+ based cardiac rehabilitation on diastolic blood pressure of patients with coronary heart disease.

**Figure 4:** Influence of Internet + cardiac rehabilitation on BMI of patients.

**Figure 5:** Influence of Internet + cardiac rehabilitation on total cholesterol of patients with coronary heart disease.

**Figure 6:** Influence of Internet-based cardiac rehabilitation on triglyceride in patients with coronary heart disease.

**Figure 7:** Funnel bias diagram of published articles.

**Table 1:** Basic data of the included articles.

Included article	Age	Sample size (IG/CG)	Intervention group	Control group	Intervention time	Evaluation indicators	Document quality
Avila et al. [9]	IG:62.2 ± 7.1 CG:63.7 ± 7.4	26/25	Internet-based home cardiac rehabilitation training	Routine nursing	3 months	①③④⑤⑥⑦⑧	B
Dale et al. [10]	IG:59.9 ± 11.8 CG:59.0 ± 10.5	61/62	Internet-based cardiac home rehabilitation training	Routine cardiac rehabilitation instruction	24 weeks	③④⑤⑥⑨⑩	A
Devi et al. [11]	IG:66.20 ± 10.06 CG:66.27 ± 8.35	36/37	Internet-based cardiac rehabilitation training	Routine nursing	6 weeks	③④⑧⑨⑩⑪	A
Dorje et al. [12]	IG:61.9 ± 8.7 CG:59.1 ± 9.4	156/156	Cardiac rehabilitation training based on mobile platform	Routine nursing	6 months	②③⑤⑥⑦⑨⑩	B
Frederix et al. [13]	IG:58 ± 9 CG:63 ± 10	34/32	Internet-based home cardiac rehabilitation training	Routine cardiac rehabilitation instruction	18 weeks	①③④⑥⑦	A
Houchen-Wolloff et al. [14]	IG:61 ± 8 CG:62 ± 10	37/23	Internet-based cardiac rehabilitation training	Routine nursing	6 months	⑧⑨⑩⑪	B
Reid et al. [15]	IG:56.0 ± 9.0 CG:56.7 ± 9.0	115/109	Internet-based cardiac rehabilitation training	Routine nursing	6 months	⑧	B
Skobel et al. [16]	IG:58 (52, 67) CG:60 (50, 65)	42/42	Internet-based cardiac rehabilitation training	Routine cardiac rehabilitation instruction	6 months	①⑤⑥⑧⑨⑩	B
Widmer et al. [17]	IG:62.5 ± 10.7 CG:63.6 ± 10.9	37/34	Cardiac rehabilitation training based on APP	Routine rehabilitation instruction	3 months	①③④⑤⑥⑦⑧	B
Zutz et al. [18]	IG:58 ± 4 CG:59 ± 12	8/5	Online cardiac rehabilitation training based on internet	Delayed intervention	12 weeks	③④⑤⑥⑦⑪	B
Fu Cong et al. [19]	IG:52.10 ± 6.44 CG:50.08 ± 12.60	54/40	Cardiac rehabilitation training based on Wechat platform	Routine coronary heart disease health education	8 weeks	③④⑥⑦⑧⑨⑩	B
Ge Cheng et al. [20]	IG:56.7 ± 10.0 CG:56.5 ± 9.0	133/133	Cardiac rehabilitation training based on wearable devices and APP	Routine health education	12 months	③④⑥⑦	B
Wang Zhao Zhao et al. [21]	IG:60.68 ± 7.09 CG:59.74 ± 8.56	28/28	Cardiac rehabilitation training based on Wechat platform	Routine cardiac rehabilitation instruction	3 months	②	B

Notes: ① The peak oxygen uptake; ② 6 min-walking experiment; ③ Systolic blood pressure; ④ Diastolic blood pressure; ⑤ BMI; ⑥ total cholesterol; ⑦ Triglyceride; ⑧ Quality of life; ⑨ Anxiety; ⑩ Depression; ⑪ self-efficacy. IG: intervention group CG: control group.

**Table 2:** Meta-analysis of Interne + based cardiac rehabilitation on other outcome indicators.

Research variable	Number of included studies	Number of study cases (T/C)	Heterogeneity test		Effect model	Meta-analysis results	
			I^2^	*P*		Effect size (95% CI)	*P*
VO2 max	4 [9, 13, 16, 17]	114/135	23%	0.27	Fixed	MD = 0.99(0.16, 1.83)	0.02
Physical activity	5 [11, 12, 18, 21]	227/229	68%	0.02	Random	SMD =0.51(0.07, 0.95)	0.02
Quality of life	4 [11, 14, 17, 19]	161/137	95%	<0.01	Random	SMD =1.34(0.13, 2.56)	0.03
Anxiety	6 [10–12, 14, 16, 19]	363/362	72%	0.01	Random	SMD = -0.34(-0.17, 0.12)	0.73
Depression	6 [10–12, 14, 16, 19]	364/365	38%	0.15	Fixed	SMD = -0.06(-0.20, 0.09)	0.45
Self-efficacy	3 [11, 14, 18]	82/67	0%	0.72	Fixed	SMD =0.50(0.17, 0.83)	0.01

## Data Availability

The labeled dataset used to support the findings of this study are available from the corresponding author upon request.
